# Identification of hsa_circ_0002024 as a prognostic competing endogenous RNA (ceRNA) through the hsa_miR_129-5p/Anti-Silencing Function 1B Histone Chaperone (ASF1B) axis in renal cell carcinoma

**DOI:** 10.1080/21655979.2021.1974650

**Published:** 2021-09-13

**Authors:** Zhe Chen, Dehua Ou, Zhuangkai Huang, Peilin Shen

**Affiliations:** a Department of Burn Surgery, The First Affiliated Hospital of Shantou University Medical College, Shantou, Guangdong Province, China; b Department of Urology, The First Affiliated Hospital of Shantou University Medical College, Shantou, Guangdong Province, China; c Department of Clinical Medicine, Shantou University Medical College, Shantou, Guangdong Province, China

**Keywords:** hsa_circ_0002024, ceRNA, hsa_miR_129-5p, ASF1b, renal cell carcinoma, bioinformatics

## Abstract

We aimed to identify novel circular RNAs (circRNAs) as prognostic competing endogenous RNAs (ceRNAs) to serve as genetic biomarkers and therapeutic targets for renal cell carcinoma (RCC). High-throughput sequencing data of circRNAs from Gene Expression Omnibus (GEO) and of microRNAs (miRNAs) and messenger RNAs (mRNAs) from The Cancer Genome Atlas (TCGA) were retrieved to identify differentially expressed RNAs (DERNAs). DEmRNAs were subjected to weighted gene coexpression network analysis (WGCNA) to identify prognostic DEmRNA (proDEmRNA) modules. Overlapping DEcircRNA-DEmiRNA and DEmiRNA-proDEmRNA interactions among the TargetScan, miRanda and RNAhybrid databases were constructed and identified. The circRNA-miRNA-mRNA ceRNA network was constructed using mutual DEmiRNAs in two interaction networks as nodes. mRNAs validated as significantly overexpressed in RCC by Oncomine, Gene Expression Profiling Interactive Analysis (GEPIA) and quantitative polymerase chain reaction (q-PCR), along with the correlative miRNAs, were used for survival analysis. Finally, a ceRNA network with 13 upregulated circRNAs, 8 downregulated miRNAs and 21 upregulated mRNAs was constructed, in which Anti-Silencing Function 1B Histone Chaperone (ASF1B) and Forkhead Box M1 (FOXM1) were considered significant by Oncomine, GEPIA and q-PCR. Survival analysis showed that ASF1B, FOXM1 and hsa_miR_1254 were significantly negatively correlated but hsa_miR_129-5p was positively correlated with overall survival time. Exploration of the ceRNA network revealed the prognostic hsa_circ_0002024/hsa_miR_129-5p/ASF1B axis. Therefore, hsa_circ_0002024 was identified as a prognostic ceRNA that might sponge hsa_miR_129-5p to regulate ASF1B and affect RCC prognosis. However, further validation is needed.

## 1 Introduction

Currently, renal cell carcinoma (RCC) is one of the most commonly diagnosed uro-oncological diseases, second only to bladder cancer [1]. RCC can be histologically classified into three major types: clear cell RCC (~80%), papillary RCC (10–15%) and chromophobe RCC (~5%) [2]. Approximately 3–5% of RCCs are familial hereditary, and up to 92% of clear cell RCCs exhibit inactivation of the Von Hippel-Lindau (VHL) gene [3,4]. Several syndromes, including VHL syndrome, hereditary clear cell RCC syndrome, etc., have been reported to increase the risk of RCC; however, the genetic association remains poorly characterized [1]. Since the 1970s, the morbidity of kidney disease has been increasing worldwide, and more than 90% of these deaths are attributed to RCC [5,6]. Although multimodal therapeutic approaches such as surgery, chemotherapy, radiotherapy and targeted therapy are available, the prognosis of RCC remains poor primarily due to the delay in diagnosis and high incidence of metastasis and recurrence [7,8]. Moreover, most patients with RCC ultimately develop drug resistance, even to targeted drugs [9]. As RCC is a histologically heterogeneous, genetically complex and prognostically poor malignant tumor, exploring the molecular mechanism of RCC to discover novel genetic biomarkers and therapeutic targets to allow its early detection and improve its prognosis is critical.

Recently, a new RNA crosstalk mechanism, named a competing endogenous RNA (ceRNA) network, has been a popular topic in cancer research. The ceRNA hypothesis, which states that messenger RNAs (mRNAs) and noncoding RNAs can communicate with each other via microRNAs (miRNAs), was first proposed by Salmena et al. in 2011 [10], and its role in cancer was further demonstrated by Karreth et al. in 2013 [11]. Typically, noncoding RNAs can interact with miRNAs to block their negative regulatory effects on mRNA expression and therefore affect the disease phenotype. As an emerging cancer biomarker and target, circular RNAs (circRNAs) can also serve as ceRNAs to regulate and control cancer progression in humans [12,13]. CircRNAs are long noncoding RNAs generated in a covalently closed-loop structure from introns, exons, untranslated regions or intergenic areas in the genome [14]. Studies have demonstrated that several circRNAs can affect the initiation and development of RCC by sponging miRNAs to regulate mRNA expression; however, the specific mechanism remains unclear [15].

In the present study, we performed a systematic study combining bioinformatics analysis using the Gene Expression Omnibus (GEO), The Cancer Genome Atlas (TCGA), Oncomine, and Gene Expression Profiling Interactive Analysis (GEPIA) databases and experimental validation by quantitative polymerase chain reaction (q-PCR) of RCC cells compared to normal kidney cells. Studies have shown that ceRNA network construction and weighted gene coexpression network analysis (WGCNA) can be used to identify RNA crosstalk networks and prognostic gene modules [16,17]. By using these approaches as our principal methods, we aimed to construct a prognostic circRNA-miRNA-mRNA ceRNA network and identify prognostic circRNA-miRNA-mRNA axes. Furthermore, multiple validation analyses were performed to identify novel circRNAs as diagnostic biomarkers and therapeutic targets for RCC.

The flow chart of the present study is shown in Figure 1.

**Figure 1.** Flow chart of the present study

GEO, Gene Expression Omnibus; TCGA, The Cancer Genome Atlas; circRNAs, circular RNAs; miRNAs, microRNAs; mRNAs, messenger RNAs; KICH, kidney chromophobe; KIRC, kidney renal clear cell carcinoma; KIRP, kidney renal papillary cell carcinoma; DEcircRNAs, differentially expressed circRNAs; DEmiRNAs, differentially expressed miRNAs; DEmRNAs, differentially expressed mRNAs; proDEmRNA, prognostic differentially expressed mRNAs; WGCNA, weighted gene coexpression network analysis; GO, Gene ontology; KEGG, Kyoto Encyclopedia of Genes and Genomes; GEPIA, Gene Expression Profiling Interactive Analysis; q-PCR, quantitative polymerase chain reaction; ceRNA, competing endogenous RNA; ASF1B, Anti-Silencing Function 1B Histone Chaperone.

## 2 Materials & Methods

### 2.1 Preprocessing of RNA sequencing data and collection of clinical information

We searched GEO (www.ncbi.nlm.nih.gov/geo/) using the keyword ‘renal cell carcinoma AND circ*’ to select high-throughput circRNA sequencing datasets of RCC published on or before 11 March 2021. The Sequence Read Archive (SRA) files and clinical information of the selected datasets were downloaded from SRA Run Selector (https://www.ncbi.nlm.nih.gov/Traces/study) for further analysis in the Linux operating system. Paired-end SRA files were divided into two single-end fastq compressed files using the Fastq-dump function in sra-tools software (version 2.10.0) [18]. After adapter trimming using Trim Galore (version 0.6.4) (www.bioinformatics.babraham.ac.uk/projects/trim_galore) and removal of low-quality reads (N base % > 5% or Q20 < 80%), the filtered reads were aligned to the hg19 reference genome/transcriptome from the UCSC Genome Browser (genome.ucsc.edu) with the BWA-MEM function in BWA software (version 0.7.17) [19]. CircRNAs were identified with CIRI software [20], annotated in the CircBase database (www.circbase.org) and finally entered into an expression matrix.

Data on miRNAs and mRNAs were retrieved from the kidney chromophobe (KICH), kidney renal clear cell carcinoma (KIRC) and kidney renal papillary cell carcinoma (KIRP) projects in the TCGA database (cancergenome.nih.gov) and analyzed with R software (version 3.6.1) [21]. We used the TCGAbiolinks package (version 2.15.3) [22] to download the high-throughput sequencing counts of miRNAs and mRNAs as well as the relevant clinical information. The miRNA and mRNA expression matrices from the above three projects were merged.

### 2.2 Differential expression analysis of circRNAs, miRNAs and mRNAs

EdgeR [23] is a package in R that can be used to identify differential expression in count-based expression data using an overdispersed Poisson model and an empirical Bayes method. It was applied for normalization and differential expression analysis of circRNAs, miRNAs and mRNAs between RCC tissues and normal kidney tissues. We filtered out RNAs with an expression count < 1, and the counts for duplicate RNAs were averaged. RNAs with a |Log (fold change (FC))|>2 and statistical p-value < 0.05 were considered differentially expressed RNAs (DERNAs) and included differentially expressed circRNAs (DEcircRNAs), differentially expressed miRNAs (DEmiRNAs) and differentially expressed mRNAs (DEmRNAs), which were further visualized in volcano plots using the ggplot2 package [24].

### 2.3 WGCNA of the DEmRNAs

WGCNA [25] is an algorithm used for the identification, summarization, membership measurement and related analysis of correlated gene modules (gene modules to gene modules or gene modules to external sample traits) and has been widely used to identify relevant genes with prognostic value in many cancers. Due to the limited quantity of DEcircRNAs and DEmiRNAs, we analyzed only DEmRNAs in RCC tumor samples using the WGCNA package in R language to evaluate gene interactions and identify coexpression modules. We calculated Pearson correlation coefficients to demonstrate the influence of the soft-thresholding power value on the scale independence and mean connectivity and subsequently chose a soft-thresholding power with a corresponding scale-free topology fit index reaching 0.95 and a corresponding maximum mean connectivity. By transforming the adjacency matrix into a topology matrix, applying the static tree cut method and setting the minimum number of genes in a module to 20, we identified coexpression gene modules and differentiated the modules by colors. Finally, the clinical information related to five prognostic factors in RCC, including tumor grade, T stage, N stage, M stage and survival time, was used to determine module-trait relationships by calculating the Pearson correlation coefficient, and the data were visualized in a heat map. With the cutoff criterion of p < 0.05, modules significantly positively related to tumor malignancy (grade and stage) and negatively related to survival time were considered prognostic DEmRNA (proDEmRNA) modules.

### 2.4 Gene ontology (GO) annotation analysis and Kyoto Encyclopedia of Genes and Genomes (KEGG) pathway enrichment analysis of the proDEmRNAs

Genes in the proDEmRNA modules were subjected to GO [26] annotation analysis and KEGG [27] pathway enrichment analysis using the clusterProfiler package [28] in R. GO annotations are classified in three components, namely, biological process (BP), cellular component (CC) and molecular function (MF), and GO terms with an adjusted p < 0.05 and a gene count >10 were considered significant. The cutoff criterion was set as an adjusted p < 0.05 in KEGG analysis to identify the pathways significantly enriched with the DEmRNAs.

### 2.5 Construction of the circRNA-miRNA-mRNA ceRNA network

TargetScan (www.targetscan.org), miRanda (www.miranda.org) and RNAhybrid (bibiserv.cebitec.uni-bielefeld.de/rnahybrid/) were used to explore the network of circRNAs, miRNAs and mRNAs. We used the local tools of the three databases to explore DEcircRNA-DEmiRNA and DEmiRNA-proDEmRNA interactions, and subsequently, the Venn web tool (bioinformatics.psb.ugent.be/webtools/Venn) was applied to identify the overlapping interactions from the three databases. Finally, using mutual DEmiRNAs in two interaction networks as nodes and considering the typical ceRNA regulation method in which a circRNA sponges an miRNA to negatively regulate the miRNA and in turn promote the expression of the target mRNA (i.e., only upregulated circRNAs, downregulated miRNAs and upregulated mRNAs were preserved in the network), we constructed a circRNA-miRNA-mRNA ceRNA network and visualized it with Cytoscape software (version 3.6.1) [29].

### 2.6 Validation of prognostic markers with Oncomine and GEPIA

To further verify the prognostic significance of the ceRNA network, we conducted comparative expression analysis of the mRNAs in Oncomine (www.oncomine.org) [30] and GEPIA (gepia.cancer-pku.cn/index.html) [31]. As Oncomine provides integrated gene expression analysis data of multiple datasets, we input ‘renal cell carcinoma vs. normal analysis’ in the filter section and selected datasets comparing mRNA expression between RCC and normal kidney tissues. The expression of prognostic mRNAs was compared between cancer tissues and normal tissues across the above datasets, and the comparison data with median ranks and combined p-values were automatically generated. The expression of prognostic mRNAs validated in Oncomine was further compared (TCGA RCC tissue vs. TCGA normal kidney tissue + Genotype-Tissue Expression (GTEx) project normal kidney tissues) with the cutoff criteria of FC > 1.5 and p-value < 0.01 in the GEPIA database for clear cell RCC, papillary RCC and chromophobe RCC, separately.

### 2.7 Cell culture

Three RCC cell lines (A498, 786-O and ACHN) and 1 normal kidney cell line (293 T) were purchased from the Chinese Academy of Sciences Shanghai Branch (China). RCC and normal kidney cells were cultured in different culture media (293 T cells in DMEM (HyClone), 786-O cells in RPMI-1640 medium (HyClone), and A498 and ACHN cells in MEM (HyClone)). All media were supplemented with 10% fetal bovine serum (Gibco, Invitrogen, USA) and cultured at 37°C in 5% CO_2_.

### 2.8 RNA isolation and q-PCR

Total RNA from 4 cell lines was isolated with TRIzol reagent (Invitrogen, USA), and cDNA was synthesized with an Evo M-MLV RT Kit with gDNA Clean for qPCR (Accurate Biotechnology, China). The expression of prognostic mRNAs validated in Oncomine and GEPIA was evaluated by a SYBR Green qPCR assay (Accurate Biotechnology, China) in an ABI 7500 Real-Time PCR System (Thermo Fisher Scientific, USA). The PCR primers used were as follows: Anti-Silencing Function 1B Histone Chaperone (ASF1B) forward, GACCTGGAGTGGAAGATCATTT; ASF1B reverse, GCCTGAAAGACAAACATGTGTC; Forkhead Box M1 (FOXM1) forward, GATCTGCGAGATTTTGGTACAC; FOXM1 reverse, CTGCAGAAGAAAGAGGAGCTAT.

### 2.9 Survival analysis

Survival analysis was performed on TCGA data for patients stratified by the expression levels of the mRNAs verified as significant by Oncomine, GEPIA and q-PCR, along with the correlative miRNAs in the ceRNA network, using the survival package (version 3.1–11) [32]. Typically, mRNAs are cancer promoters and are negatively correlated with survival outcomes in the ceRNA network, while miRNAs have the opposite relationship. Therefore, we set p < 0.05 as the significance criterion to identify negative prognostic mRNAs and positive prognostic miRNAs. CircRNAs that sponged positive prognostic miRNAs to upregulate negative prognostic mRNAs in the ceRNA network were considered negative prognostic factors.

## 3 Results

We analyzed data from GEO and TCGA by differential expression analysis and WGCNA to identify DEcircRNAs, DEmiRNAs, and proDEmRNA modules, from which a circRNA-miRNA-mRNA ceRNA network was constructed. Via comparative mRNA expression analysis of the Oncomine and GEPIA databases, q-PCR in RCC and normal kidney cell lines, and survival analysis in TCGA, we validated a prognostic circRNA-miRNA-mRNA axis and identified a novel circRNA as a prognostic ceRNA in RCC.

### 3.1 Identification of DEmRNAs, DEmiRNAs, and DEcircRNAs

The GEO search identified 31 records, among which only one dataset, GSE108735 (www.ncbi.nlm.nih.gov/geo/query/acc.cgi?acc=GSE108735), contained second-generation circRNA sequencing data (Table 1). In addition, mRNA data of 1019 samples (891 RCC and 128 normal kidney tissues) and miRNA data of 1031 samples (901 RCC and 130 normal kidney tissues) were retrieved from TCGA. After normalization and differential expression analysis of expression matrixes with the EdgeR package, 113 DEcircRNAs (all upregulated), 56 DEmiRNAs (upregulated, 39; downregulated, 17) and 3807 DEmRNAs (upregulated, 2865; downregulated, 942) were identified and visualized in volcano plots (Figure 2).

**Table 1.** Clinical characteristics of GSE108735

sample	GEO Accession	Age	gender	tumor_stage
normal	GSM2912685	63	male	\
	GSM2912686	64	male	\
	GSM2912687	53	female	\
	GSM2912688	60	male	\
	GSM2912689	53	female	\
	GSM2912690	60	male	\
	GSM2912691	61	male	\
renal cell carcinoma	GSM2912692	63	male	T1N0M0
	GSM2912693	64	male	T1N0M0
	GSM2912694	53	female	T1bN0M0
	GSM2912695	60	male	T1bN0M0
	GSM2912696	53	female	Unknow
	GSM2912697	60	male	T1N0M0
	GSM2912698	61	male	T1N0M0

**Figure 2.** Identified DERNAs from GEO and TCGA. (a) 113 upregulated differentially expressed circular RNAs were identified from GSE108735. (b) 56 differentially expressed microRNAs with 39 upregulated ones and 17 downregulated ones were identified from The Cancer Genome Atlas (TCGA). (c) 3807 differentially expressed messenger RNAs with 2865 upregulated ones and 942 downregulated ones were identified from TCGA

### 3.2 WGCNA, GO annotation analysis and KEGG pathway analysis

A total of 889 RCC patients with 3807 identified DEmRNAs were included for WGCNA. After calculation of the soft-thresholding power, a threshold power of 3 was found to correspond with a scale-free topology fit index reaching 0.95 and the maximum mean connectivity and was therefore set as the cutoff threshold (Figure 3a). By applying the cutoff threshold and performing WGCNA, we identified 11 gene coexpression modules with more than 20 genes each (Figure 3b). Module-trait relationships were identified and visualized; the red module, with 50 genes, was considered a proDEmRNA module due to its significant positive correlation with tumor malignancy (p_Grade_ = 1e-26, p_T stage_ = 3e-22, p_N stage_ = 9e-13, p_M stage_ = 4e-25) and negative correlation with survival time (p_Survival time_ = 5e-6) (Figure 3c).

**Figure 3.** WGCNA of the DEmRNAs. (a) Analysis of network topology for different soft-thresholding powers. (b) 11 coexpression gene modules of more than 20 genes each were demonstrated in the clustering dendrogram with assigned module colors. (c) In the correlation of mRNA coexpression network modules with clinical prognostic factors of RCC, red module had a significant positive correlation with tumor malignancy (grade and stage) and negative correlation with survival time

The proDEmRNAs were highly related to the cell cycle pathway in both the GO and KEGG analyses. In the GO analysis, although none of the significantly enriched MF terms contained more than 10 genes, the proDEmRNAs were enriched mainly in 18 BP terms related to the cell cycle (nuclear division, organelle fission, chromosome segregation, etc.) and classified in three relative CC terms (chromosome, spindle and microtubule) (Figure 4(a,b)). The cell cycle was also the most enriched pathway in the KEGG analysis (Figure 4c).

**Figure 4.** GO annotation analysis and KEGG pathway enrichment analysis of proDEmRNAs. (a)Terms enriched in biological processes of Gene ontology (GO) enrichment analysis were as follows: nuclear division, organelle fission, mitotic nuclear division, chromosome segregation, regulation of mitotic nuclear division, regulation of nuclear division, sister chromatid segregation, nuclear chromosome segregation, mitotic sister chromatid segregation, regulation of mitotic cell cycle phase transition, cell cycle checkpoint, cytokinesis, regulation of cell cycle phase transition, cell cycle G2/M phase transition, positive regulation of cell cycle process, negative regulation of mitotic cell cycle, negative regulation of cell cycle process, positive regulation of cell cycle. (b) Terms enriched in cellular components of GO enrichment analysis were as follows: condensed chromosome, spindle, microtubule. (c) Pathways enriched in Kyoto Encyclopedia of Genes and Genomes analysis were cell cycle, oocyte meiosis and progesterone-mediated oocyte maturation

### 3.3 CircRNA-miRNA-mRNA ceRNA network construction

After interaction analysis using TargetScan, miRanda and RNAhybrid, DEcircRNA-DEmiRNA and DEmiRNA-proDEmRNA interaction networks in the three databases were constructed. The DEcircRNA-DEmiRNA networks contained 1174 interactions in TargetScan, 1532 interactions in miRanda and 307 interactions in RNAhybrid. The DEmiRNA-proDEmRNA networks contained 871 interactions in TargetScan, 1136 interactions in miRanda and 305 interactions in RNAhybrid. Subsequently, 39 overlapping DEcircRNA-DEmiRNA interactions and 120 overlapping DEmiRNA-proDEmRNA interactions were identified by Venn diagram analysis of the three databases (Figure 5). Using mutual DEmiRNAs in two overlapping interaction networks as nodes, we constructed the relationships among 26 circRNAs, 17 miRNAs and 25 mRNAs. Finally, after removing 9 upregulated miRNAs and 17 unconnected nodes (13 circRNAs and 4 mRNAs), we retained 13 upregulated circRNAs, 8 downregulated miRNAs and 21 upregulated mRNAs to construct the ceRNA network (Figure 6).

**Figure 5.** Overlapping interactions derived from the intersection analysis of TargetScan, miRanda and RNAhybird. (a) Networks of differentially expressed circular RNAs (DEcircRNAs) to differentially expressed microRNAs (DEmiRNAs) contained 1174 interactions in TargetScan, 1532 interactions in miRanda and 307 interactions in RNAhybird. A total of 39 overlapping interactions of DEcircRNAs to DEmiRNAs were identified with Venn intersection analysis. (b) Networks of DEmiRNAs to prognostic differentially expressed messenger RNAs (proDEmRNAs) contained 871 interactions in TargetScan, 1136 interactions in miRanda and 305 interactions in RNAhybird. A total of 120 overlapping interactions of DEmiRNAs to proDEmRNAs were identified with Venn intersection analysis

**Figure 6.** The circRNA-miRNA-mRNA ceRNA network

The competing endogenous RNA network was constructed with 13 upregulated circular RNA RNAs, 8 downregulated microRNAs and 21 upregulated messenger RNAs, in which the identified prognostic axis of hsa_circ_0002024/hsa_miR_129-5p/Anti-Silencing Function 1B Histone Chaperone (ASF1B) is marked with a dashed ellipse.

### 3.4 Comparative mRNA expression, q-PCR and survival analyses

Fifteen comparative analysis datasets were found in Oncomine, and the expression of 21 mRNAs was assessed in these datasets. Eighteen mRNAs showed no statistically significant difference between RCC and normal kidney samples, while three – ASF1B (p = 0.012), Ribonucleotide Reductase Regulatory Subunit M2 (RRM2) (p = 0.002) and FOXM1 (p = 0.024) – were considered significant (Figure 7). The expression data of the three significant mRNAs was further presented as boxplots in GEPIA, which showed that only ASF1B and FOXM1 were significantly overexpressed in all 3 subtypes of RCC (Figure 8). Figure 9 confirms the higher mRNA abundance of ASF1B and FOXM1 in RCC cell lines (ASF1B in A498, 786-O and ACHN cells; FOXM1 in 786-O and ACHN cells) than in the normal kidney cell line 293 T.

**Figure 7.** Pooled comparative analysis of the mRNA expression in Oncomine database

* The rank for a gene is the median rank for that gene across each of the analyses. †The p-Value for a gene is its p-value for the median-ranked analysis.1. Hereditary Clear Cell Renal Cell Carcinoma vs. Normal; Beroukhim Renal, Cancer Res, 20092. Non-Hereditary Clear Cell Renal Cell Carcinoma vs. Normal; Beroukhim Renal, Cancer Res, 20093. Clear Cell Sarcoma of the Kidney vs. Normal; Cutcliffe Renal, Clin Cancer Res, 20054. Clear Cell Renal Cell Carcinoma vs. Normal; Gumz Renal, Clin Cancer Res, 20075. Chromophobe Renal Cell Carcinoma vs. Normal; Higgins Renal, Am J Pathol, 20036. Clear Cell Renal Cell Carcinoma vs. Normal; Higgins Renal, Am J Pathol, 20037. Granular Renal Cell Carcinoma vs. Normal; Higgins Renal, Am J Pathol, 20038. Papillary Renal Cell Carcinoma vs. Normal; Higgins Renal, Am J Pathol, 20039. Chromophobe Renal Cell Carcinoma vs. Normal; Jones Renal, Clin Cancer Res, 200510. Clear Cell Renal Cell Carcinoma vs. Normal; Jones Renal, Clin Cancer Res, 200511. Papillary Renal Cell Carcinoma vs. Normal; Jones Renal, Clin Cancer Res, 200512. Clear Cell Renal Cell Carcinoma vs. Normal; Lenburg Renal, BMC Cancer, 200313. Chromophobe Renal Cell Carcinoma vs. Normal; Yusenko Renal, BMC Cancer, 200914. Clear Cell Renal Cell Carcinoma vs. Normal; Yusenko Renal, BMC Cancer, 200915. Papillary Renal Cell Carcinoma vs. Normal; Yusenko Renal, BMC Cancer, 2009

**Figure 8.** Box-plots of mRNA expression between RCC and normal kidney in GEPIA database

The message RNAs expression of Anti-Silencing Function 1B Histone Chaperone (ASF1B), Ribonucleotide Reductase Regulatory Subunit M2 (RRM2) and Forkhead Box M1 (FOXM1) between renal cell carcinoma (RCC) and normal kidney in Gene Expression Profiling Interactive Analysis (GEPIA) database using data from The Cancer Genome Atlas (TCGA) and Genotype-Tissue Expression (GTEx) was demonstrated. Fold change > 1.5 and p value < 0.01 were considered significant and only ASF1B and FOXM1 showed significant overexpression in clear cell RCC, papillary RCC and chromophobe RCC.

**Figure 9.** Relative expression of ASF1B and FOXM1 in q-PCR

In comparison with normal kidney cells 293 T, Anti-Silencing Function 1B Histone Chaperone (ASF1B) was with higher message RNA (mRNA) abundance in A498, 786-O and ACHN, and Forkhead Box M1 (FOXM1) was with higher mRNA abundance in 786-O and ACHN. *, p < 0.05; **, p < 0.01; ***, p < 0.001.

Survival curves for patients stratified by the expression levels of two significant mRNAs and four correlative miRNAs (hsa_miR_129-5p, hsa_miR_193a-5p, hsa_miR_1254 and hsa_miR_4433a-5p) in the ceRNA network were constructed with R software. The survival analyses for mRNAs included 889 RCC patients and the survival analyses of miRNAs involving 860 RCC patients were conducted. While both mRNAs were significantly negatively correlated with overall survival time (all p < 0.001), hsa_miR_129-5p was the only positive prognostic miRNA (p = 0.0212) (Figure 10). Therefore, we explored the circRNA-miRNA-mRNA interactions in the ceRNA network and identified hsa_circ_0002024 as a negative prognostic factor that acts by sponging and suppressing hsa_miR_129-5p to promote ASF1B expression in RCC. The prognostic hsa_circ_0002024/hsa_miR_129-5p/ASF1B axis is marked with a dashed ellipse in Figure 6.

**Figure 10.** Survival analysis of the significant mRNAs and correlative miRNAs in the ceRNA network

Anti-Silencing Function 1B Histone Chaperone (ASF1B), Forkhead Box M1 (FOXM1) and hsa−miR−1254 had significant negative correlations with overall survival time, while hsa_miR_129-5p had significant positive correlation with overall survival time.

## 4 Discussion

As mRNAs encode proteins that participate in various BPs, any factor that interferes with the normal expression of mRNAs can possibly cause abnormal cell proliferation and differentiation and eventually lead to carcinogenesis. MiRNAs bind to specific 3′-untranslated regions (3′-UTRs) of mRNA transcripts to cause mRNA degradation and regulate downstream signaling pathways [33,34]. As a newly discovered RNA species, circRNAs are considered to have multiple functions, such as protein translation, participating in circRNA–protein interactions and, most importantly, acting as ceRNAs [35]. The structural stability of the closed loop of circRNAs provides natural resistance to exoribonucleases, which makes circRNAs highly stable in the cytoplasm [36]. Given their natural stability, circRNAs have been described as reliable potential regulators in multiple cancers and could possibly serve as a promising biomarker and novel therapeutic target [37].

The ceRNA hypothesis describes an intricate interplay among mRNAs, miRNAs and noncoding RNAs such as long-noncoding RNAs, pseudogenes and circRNAs [38], in which circRNAs function as a sponge-like endogenous competitive factor for miRNAs to regulate the expression of mRNAs and thereby contribute to tumor proliferation and invasion [39,40]. Unlike miRNAs, the regulatory mechanism through which circRNAs function as miRNA sponges remains unclear, despite numerous studies [41]. Many miRNAs (miR-216b [42], miR-488 [43], miR-193a-3p and miR-224 [44]) and circRNAs (circ_0001368 [45], circ_0039569 [46] and hsa_circ_0054537 [47]) have been suggested to be crucial for the proliferation and invasion of RCC cells.

This systematic study combining bioinformatics analysis and experimental validation was performed to identify novel prognostic circRNAs as diagnostic biomarkers and therapeutic targets for RCC. We used differential expression analysis to identify DERNAs and then applied WGCNA to identify the red proDEmRNA module. A ceRNA network was constructed among the DEcircRNAs, DEmiRNAs and red module, in which two mRNAs, ASF1B and FOXM1, were validated as significant by Oncomine, GEPIA and q-PCR. The two validated mRNAs, along with the four correlative miRNAs (hsa_miR_129-5p, hsa_miR_193a-5p, hsa_miR_1254 and hsa_miR_4433a-5p) in the ceRNA network, were used for survival analysis to identify the positive survival-related mRNAs (ASF1B and FOXM1) and negative survival-related miRNA (hsa_miR_129-5p). Based on the interactions in the ceRNA network, the hsa_circ_0002024/hsa_miR_129-5p/ASF1B axis was identified; thus, hsa_circ_0002024 was revealed to be the prognostic ceRNA in RCC.

ASF1B, a subtype of ASF1, encodes a histone H3-H4 chaperone protein, which is the substrate of the tousled-like kinase family of cell cycle-regulated kinases and may catalyze the assembly and disassembly of the nucleosome structure of chromatin. When the nucleosome structure of chromatin is not appropriately modulated, diseases such as cancers occur [48,49]. Studies have demonstrated that ASF1 regulates chromatin function and promotes cancer development, especially the ASF1B subtype, which has been reported as a promoter of multiple cancers [50]. Both ASF1B and hsa_miR_129-5p have been demonstrated to contribute to the same cancers, for example, breast cancer [51,52], prostate cancer [53,54] and RCC [50,55], although no interactions have been established. However, both Zhou et al. [50] and Chiang et al. [55] found that ASF1B and hsa_miR_129-5p were involved in AKT signal transduction pathway activation in RCC. The AKT signal transduction pathway regulates many cellular processes, such as survival, proliferation, growth, metabolism, angiogenesis and metastasis [56], and its hyperactivation has been abundantly demonstrated to be involved in the initiation, progression, and drug resistance of many cancers; thus, it is a therapeutic target in cancer [57]. Collectively considering the evidence that the AKT pathway plays a critical role in malignant tumors with the results of the present study, we can hypothesize that hsa_circ_0002024 sponges hsa_miR_129-5p to regulate ASF1B and increase the occurrence, metastasis and fatality rate of RCC via the AKT pathway.

This study has several limitations, such as methodological bias, data heterogeneity, experimental simplicity and lack of in vivo experimental validation. These limitations contribute to the differences in the results and impact the reliability of this study.

## 5 Conclusion

In summary, we identified hsa_circ_0002024 as a novel diagnostic biomarker and therapeutic target ceRNA. Hypothetically, hsa_circ_0002024 can sponge hsa_miR_129-5p to impact its binding to ASF1B, thereby resulting in overexpression of ASF1B and eventually leading to cell cycle dysregulation and an aberrant nucleosome structure in chromatin. These events play a role in the occurrence and development of RCC, possibly via the AKT signal transduction pathway. However, further biological studies are necessary to verify our research findings.

## Supplementary Material

Supplemental Material

## Data Availability

The datasets analyzed for this study can be found in the GEO database (www.ncbi.nlm.nih.gov/geo), TCGA database (cancergenome.nih.gov), Oncomines database (www.oncomine.org) and GEPIA database (gepia.cancer-pku.cn).

## Research highlights

1. We identified the novel hsa_circ_0002024/hsa_miR_129-5p/ASF1B ceRNA axis for RCC.
2. hHsa_circ_0002024 might sponge hsa_miR_129-5p to promote ASF1B via the AKT pathway.
3. hHsa_circ_0002024 was verified as a prognosticator both in silicon and in vitro.

All authors have read and approved this manuscript.
